The article "Seed germination ecology of Conyza stricta Willd. and implications for management" was retracted in 2024. Reasons: a conflict of interest; concerns about the peer review; concerns about the authorship.

# Seed germination ecology of *Conyza stricta* Willd. and implications for management

**DOI:** 10.1371/journal.pone.0244059

**Published:** 2020-12-29

**Authors:** Safdar Ali, Fakhar Din Khan, Rehmat Ullah, Rahmat Ullah Shah, Saud Alamri, Maeesh AlHarthi, Manzer H. Siddiqui

**Affiliations:** 1 Directorate of Land Reclamation, Government of Punjab, Lahore, Pakistan; 2 Soil and Water Testing Laboratory for Research, Dera Ghazi Khan, Pakistan; 3 Department of Soil Science, Faculty of Agricultural Sciences and Technology, Bahauddin Zakariya University, Multan, Pakistan; 4 Department of Botany and Microbiology, College of Science, King Saud University, Riyadh, Saudi Arabia; Harran University, TURKEY

## Abstract

Numerous cropping systems of the world are experiencing the emergence of new weed species in response to conservation agriculture. *Conyza stricta* Willd. is being a newly emerging weed of barley-based cropping systems in response to conservational tillage practices. Seed germination ecology of four populations (irrigated, rainfed, abandoned and ruderal habitats) was studied in laboratory and greenhouse experiments. The presence/absence of seed dormancy was inferred first, which indicated seeds were non-dormant. Seed germination was then recorded under various photoperiods, constant and alternating day/night temperatures, and pH, salinity and osmotic potential levels. Seedling emergence was observed from various seed burial depths. Seeds of all populations proved photoblastic and required 12-hour light/dark period for germination. Seeds of all populations germinated under 5–30°C constant temperature; however, peak germination was recorded under 17.22–18.11°C. Nonetheless, the highest germination was noted under 20/15°C alternating day/night temperature. Ruderal and irrigated populations better tolerated salinity and germinated under 0–500 mM salinity. Similarly, rainfed population proved more tolerant to osmotic potential than other populations. Seeds of all populations required neutral pH for the highest germination, whereas decline was noted in germination under basic and alkaline pH. Seedling emergence was retarded for seeds buried >2 cm depth and no emergence was recorded from >4 cm depth. These results add valuable information towards our understanding of seed germination ecology of *C*. *stricta*. Seed germination ability of different populations under diverse environmental conditions suspects that the species can present severe challenges in future if not managed. Deep seed burial along with effective management of the emerging seedlings seems a pragmatic option to manage the species in cultivated fields. However, immediate management strategies are needed for rest of the habitats.

## Introduction

*Conyza* genus belonging to Asteraceae family includes 80–100 species, mainly distributed in tropical and sub-tropical regions of the world [1]. Most of the *Conyza* species are winter-annuals and native to North America. *Conyza* species are distributed in several cropping systems and exert significant yield and quality losses in field crops [2]. These species could tolerate adverse environmental conditions; thus, are capable of becoming troublesome under changing climate. *Conyza canadensis*, *C*. *bonariensis* and *C*. *sumatrensis* are the main species of the genus, widely studied for their seed germination biology and seedling emergence characteristics under various environmental conditions [3–7]. *Conyza canadensis* is distributed over a large area in North America and Europe [8, 9].

Tillage is exploited as a weed management tool in conservation agriculture [10]. Increasing evidences of herbicide resistance has forced researchers to find alternatives of herbicides, and tillage is being used to manage weeds [11]. Reducing soil seed bank is the long term goal of tillage in conservation agriculture. Several studies have been conducted to infer the impact of tillage practices on soil seed bank and contrasting results have been reported. Studies have reported an increase [12], decrease [13] or no impact [14] of tillage on soil seed bank. Nonetheless, various studies on seed germination biology of weed species have indicated that tillage can be used to reduce soil seed bank in long run [15–17]. Moreover, vertical distribution of seeds in the soil is also controlled by the tillage [10]. The altered tillage practices in conservation agriculture are resulting in weed flora shifts in several regions of the world [18]. No or reduced tillage favor some weeds, while suppress other weeds [12]. Thus, it is clear that altered tillage practices are resulting in weed flora shifts, subsequently giving rise to new weed outbreaks.

*Conyza stricta* (erect horseweed), a member of the *Conyza* genus is recently being observed in several cropping systems of the world under conservation agricultural practices [19, 20]. It is a winter annual growing ~1.1 m [21]. The species grows within an altitude range of 500–2000 m. The plant is used for several medicinal purposes [22]. However, the ‘weed’ status has rarely been given to the species. Recent climate changes and greenhouse gases’ emission have forced agricultural production towards conservation agriculture practices [23, 24]. Rapid flip between conventional and conservational tillage practices have resulted in the emergence of new weed species [10, 20, 25]. However, the knowledge regarding germination biology of such species is insufficient. Newly emerging weed species are difficult to control due to lack of seed germination biology knowledge. Control over seed germination is the first step for successful management of weed species.

Several environmental cues, including light, temperature, soil salinity, pH and water potential of the soil alter seed germination and seedling emergence of plant species [3, 26–28]. The seeds of *Conyza* species are positively photoblastic [2, 29], and rarely emerge from deep burial depths [16, 17, 30]. Seed dormancy is an important biological trait influencing the germination and persistence of weed species. *Conyza* species have no or low dormancy [5], while some studies have reported high seed dormancy in these species [31]. Seeds of *Conyza* species become dormant under adverse environmental conditions and resume germination once environmental conditions become suitable [32].

Temperature is an important factor controlling seed germination since it impacts moisture uptake, enzymatic reactions and physiological processes necessary for germination [33]. *Conyza* species, being winter annuals are known to germinate under 20 and 30°C, with 20°C as optimum temperature for seed germination [2, 5, 7, 9, 30, 34]. However, seed germination under higher temperature is also observed indicating that these species can germinate round the year [7, 29, 34].

Seeds of *Conyza* are photoblastic and emergence from the upper soil layers. Deep buried seeds of *Conyza* species are unable to emerge because of insufficient light availability [7, 32]. *Conyza* species are less persistent in the soil due to absence of seed dormancy; however, high fecundity enables them to invade numerous habitats. Seed viability of non-germinating seeds is rapidly lost due non-dormant nature [5]. Seedling recruitment helps weed species to get established in new habitats [35]. The knowledge of magnitude and timing of seedling emergence can be used for successful management of weed species under field conditions [36, 37]. Zambrano-Navea et al. [38] have predicted seedling emergence and population dynamics of *C*. *bonariensis* [39]. However, such models are unavailable for *C*. *stricta* due to missing knowledge on seed germination biology.

*Conyza* species are evolving resistance to several herbicides globally [11]. Nonetheless, herbicides are frequently used in conservation agriculture, which could also lead towards evolution of herbicide resistance. Chemical weed control is a promising option to manage *Conyza* species [29, 40]. However, increasing cases of herbicide resistance will render chemical control inefficient. Thus, alternative, eco-friendly weed management option are needed for the management of *Conyza* species. Tillage practices in conservation agriculture can be exploited to manage these species. However, sound knowledge of seed germination biology is required to use tillage as a management tool.

Seed germination ecology of *C*. *stricta* is unknown, which makes it difficult to control under field conditions. The 10–25°C is regarded as temperature range for the germination of *Conyza* species, excluding *C*. *stricta* [4]. However, optimum and upper and lower limits of temperature are unknown for *C*. *stricta* [5]. Light is not an inherent requirement for seed germination of *C*. *canadensis* [41]. However, some other studies reported that *Conyza* species are photoblastic [4, 42]. Plenty of knowledge exists on the biology [6] and emergence [2, 4, 31, 34, 43, 44] of *C*. *canadensis*, *C*. *bonariensis* and *C*. *sumatrensis*. However, information is lacking on seed germination biology of *C*. *stricta*, resulting in poor understanding and control of this weed.

The current study was conducted to infer the impact of different environmental factors on seed germination of different populations of *C*. *stricta*. Studying germination characteristics from different sites of origin provides better understanding of germination biology [30]. Therefore, we included four different populations in the study stemming from different habitats to possibly cover the full distribution range. We were interested to infer; i) the environmental conditions favoring seed germination of *C*. *stricta*, ii) whether population stemming from different habitats exhibit differences in seed germination biology, iii) what is the tolerance level of different populations to salinity and osmotic potential and iv) if increasing seed burial depth could suppress the seedling emergence. The results would improve the understanding on seed germination biology and help in the management of the species.

## Materials and methods

### Seed collection

Seeds of *Conyza stricta* were collected from four different habitats to possibly cover full distribution range of habitats. Conservation agriculture is being practiced in irrigated and rainfed areas, where species has recently emerged as weed [19, 45]. Therefore, seeds were collected from irrigated, rainfed, abandoned and ruderal habitats. The background information on the seed collection sites is presented in Table 1. Seed were collected from 40 mother plants randomly, brought to laboratory, dried and stored in glass jars at 20°C until use. Soil samples were collected from the seed collection sites and analyzed according to Farooq et al. [17]. The soil properties of the seed collection sites are presented in Table 2. The soils of irrigated and ruderal population were moderately saline, whereas rainfed and abandoned habitats were non-saline. Seed collection did not require any permission and no endangered species were involved in the study.

**Table 1:** Background information on the seed collection sites and some plant traits.

Habitat	Latitude °N	Longitude °E	Tillage practice	Irrigation	Plant height (cm)	Seeds plant^-1^
Irrigated	30.419624	72.302677	Zero tillage	Yes	45.68	2921
Rainfed	30.955700	70.915614	Conservational tillage	No	34.32	1633
Abandoned	30.544327	72.125319	-	No	36.87	1743
Ruderal	30.093521	72.975835	-	No	31.23	1609

**Table 2:** Soil properties of seed collection sites.

Habitat	CaCO_3_ (%)	OM (%)	pH	EC (mS/m)	Clay (%)	Sand (%)	Silt (%)	P (ppm)
Irrigated	46.00	2.55	8.41	337.20	57.70	22.30	20.00	51.91
Rainfed	22.67	0.69	7.92	109.40	25.20	47.30	27.50	28.58
Abandoned	74.58	1.24	7.75	98.00	47.70	22.30	30.00	41.92
Ruderal	10.44	1.12	7.64	490.00	31.10	46.40	22.50	30.73

OM = organic matter, P = phosphorus, EC = electrical conductivity.

## Experimental details

Seven different experiments (six laboratory and one greenhouse) were conducted to infer the seed germination ecology of *C*. *stricta*. Environmental cues and their respective treatments/levels included in the experiments are summarized in Table 3. Seed dormancy test was conducted to infer dormancy status of the seeds, which indicated no dormancy. Therefore, no seed dormancy release treatments were required for germination tests. Seed germination was recorded under three different light/dark durations to infer the impact of photoperiod. Germination was evaluated under ten constant and four alternating day/night temperatures. Germination was noted under fourteen NaCl salinity and fifteen osmotic potentials. Salinity and osmotic potential solutions were prepared following Chauhan et al. [46] and Michel and Kaufmann [47], respectively. Seeds of all populations were germinated under 10 pH levels, representative of neutral, acidic and alkaline pH. Seedling emergence was observed from 13 different seed burial depths.

**Table 3:** The details of environmental cues and their levels used to study the seed germination biology of *Conyza stricta* Wildd.

Environmental factor	Levels/treatments
Light/dark duration (hours)	0, 12, 24
Temperature (°C)	5, 10, 15, 20, 25, 30, 35, 40, 45, 50
Day/night varying temperature (°C)	15/10, 20/15, 15/15, 20/10
Salinity levels (mM NaCl)	0, 25, 50, 100, 150, 200, 250, 300, 350, 400, 450, 500, 550, 600
Osmotic potentials (-MPa)	0, 0.1, 0.2, 0.3, 0.4, 0.5, 0.6, 0.7, 0.8, 0.9, 1, 1.1, 1.2, 1.3, 1.4
pH levels	3, 4, 5, 6, 7, 8, 9, 10, 11, 12
Seed burial depth (cm)	0, 1, 2, 3, 4, 5, 6, 7, 8, 9, 10, 11, 12

### Experimental design

All experiments were conducted separately and laid out in a factorial design. The populations were considered as main factor, whereas levels/treatments were regarded as sub-factor. All experiments were repeated over time. Fifty seeds were germinated in Petri dish and three dishes were considered as a single replication. All experiments had five replications.

### Experimental procedure

Seed germination was recorded in 90-mm diameter Petri dishes. Two layers of Whatman no. 1 filter paper were placed at the bottom of dishes. Fifty seeds were placed on filter paper. The filter paper was moistened with 6 ml distilled water or treatment solution according to the experiments (Table 3). The Petri dishes were incubated under 20/15°C alternating day/night temperature except for the constant temperature experiment. Similarly, the light duration in incubators was adjusted to 12-hour day/night cycle except for the light/dark experiment. Petri dishes of complete dark treatment were wrapped in four layers of aluminum foil to exclude the impacts of light. The dishes were sealed with paraffin film to avoid moisture loss through evaporation. Seed germination was recorded 30 days after the start of experiments. The non-germinating seeds were tested for viability by Tetrazolium test [48]. Finally, seed germination percentage was computed for each treatment and adjusted for viable, non-germinating seeds according to Weller et al. [49]. Viability adjusted seed germination percentage was used for statistical analysis and interpretation of the results.

### Statistical analysis

Normality in the data was tested by Shapiro-Wilk normality test [50], which indicated a normal distribution. Therefore, statistical analyses were performed on original data. The data of light/dark and alternating day/night temperature experiments were analyzed by Analysis of Variance (ANOVA) technique [51]. Two-way ANOVA was used to infer the significance in the data of light/dark and alternating temperature experiments. Least significant difference test at 5% probability was used to separate the means where ANOVA denoted significant differences. Gaussian model was fitted to the data of constant temperature, pH and seed burial experiments. The model was;

$$G=a\times e\left[‐0.5‐{\left\{\left(x-b\right)/c\right\}}^{2}\right]$$

Here, “a” = the highest viability adjusted seed germination % or seedling emergence %, “b” = environmental condition under which the highest germination or seedling emergence was recorded and “c” = width of the “bell”.

The data of salinity and osmotic potential experiments were analyzed by a three-parameter sigmoid model. The model was:

$$G=G_{max}/\left(1+e\left[‐x‐T_{50}\right)/G_{rate}\right]$$

Here; G = viability adjusted seed germination %, G_max_ = viability adjusted maximum germination %, T_50_ = environmental condition required to retard 50% of maximum germination, and G_rate_ = slope. The ANOVA was performed on SPSS version 21.0 [52], whereas SigmaPlot version 13.0 was used to fit the Gaussian and sigmoid models.

## Results and discussion

### Light/dark periods

Different light/dark durations have significant impact on seed germination of all populations. Seeds of all population were purely photoblastic. Overall, the highest germination was recorded for irrigated population under 12-hour light/dark period, whereas complete dark resulted in the lowest germination of all populations (Fig 1).

**Fig 1:** The influence of different light/dark durations on seed germination *Conyza stricta* Willd. The vertical bars present standard errors of means (n = 10). Any to means sharing same letter are statistically non-significant (p>0.05). LDS 0.05 = 4.36.

There were slight differences in seed germination of tested populations and irrigated population had higher germination. These differenced are linked to the frequent disturbance faced by irrigated areas as seed collection site was under agricultural practices (Table 1). Several earlier studies have confirmed that seeds of *Conyza* species are purely photoblastic and require 12-hour light/dark duration for germination [4, 7, 30, 42]. This behavior of the seeds can be exploited for the management of the species in agricultural habitats. Seed burial to a depth where light did not reach to the seeds can be a successful management strategy against the species. This hypothesis is also supported by the results of seed burial experiment where deep burial completely retarded seed germination.

### Constant and alternating day/night temperature

Different constant temperatures influenced seed germination of all populations. Seeds were able to germinate under a wider range of constant temperatures (5–30°C). Germination was initially increased with increasing temperature up to 20°C and then a sudden decline was noted for all populations (Fig 2). The highest and the lowest germination potential was recorded for irrigated and ruderal populations, respectively (Table 4). Optimum temperature for the highest seed germination of the populations ranged from 17.22 to 18.11°C.

**Fig 2:** The influence of different constant temperatures on seed germination of *Conyza stricta* Willd. The vertical bars present standard errors of means (n = 10).

**Table 4:** Effect of different environmental conditions on seed germination of different populations of *Conyza stricta* Willd. modeled with three parametric Gaussian equation.

Population	G_max_	T_max_	G_rate_	R^2^
**Constant temperatures**				
Irrigated	96.95±2.79	17.22±0.22	6.61±0.21	0.99
Rainfed	89.53±2.87	17.31±0.23	6.40±0.22	0.99
Abandoned	88.75±2.37	17.73±0.19	6.28±0.18	0.99
Ruderal	75.72±4.19	18.11±0.39	6.11±0.48	0.97
**pH**				
Irrigated	86.19±3.93	7.07±0.12	2.29±0.11	0.95
Rainfed	91.09±3.64	7.03±0.08	1.91±0.07	0.97
Abandoned	91.96±3.33	7.32±0.09	2.17±0.08	0.96
Ruderal	90.97±3.54	7.34±0.10	2.38±0.11	0.96
**Seed burial depth**				
Irrigated	85.78±6.21	1.77±0.12	1.44±0.13	0.94
Rainfed	88.23±4.69	1.72±0.06	1.03±0.05	0.97
Abandoned	91.15±4.86	1.62±0.06	1.01±0.05	0.96
Ruderal	86.51±3.70	1.69±0.04	0.99±0.05	0.98

Parameter estimates: G_max_ = maximum germination (%), T_max_ = respective environmental conditions to achieve the maximum germination (days), G_rate_ = width of the bell of three parametric Gaussian function fitted to model the germination of different populations of Erect horseweed. R^2^ represents the model goodness of fit.

Several necessary enzymes for seed germination are activated by temperature [26]. Decreasing seed germination with increasing temperature can be linked to the winter annual nature of the species [21, 22]. Slight differences among seed germination of the tested populations are due to the morphological/genetic variations. Several studies have reported that populations of the same species differ in their temperature requirement due to morphological variations [17, 53–57]. However, no strong evidence is available for genetic effect on seed germination of different populations of the same species.

Seed germination of all populations was affected by different alternating day/night temperatures. The 20/15°C resulted in the highest germination of tested populations, while 15/10°C resulted in the lowest germination (Fig 3). These results indicate that day/night variation under natural conditions strongly affect germination of weed species. Several studies on seed germination of weed species have reported better germination under alternating compared to constant temperature.

**Fig 3:** The influence of different alternating day/night temperatures on seed germination of *Conyza stricta* Willd. The vertical bars present standard errors of means (n = 10). Any to means sharing same letter are statistically non-significant (p>0.05). LDS 0.05 = 4.87.

*Conyza* species being winter annuals are known to germinate under 20 and 30°C, with 20°C as optimum temperature germination [2, 5, 7, 9, 30, 34]. However, seed germination under higher temperature is also observed indicating that the species can germinate round the year [7, 29, 34].

### Salinity levels

Different salinity levels strongly affected seed germination of different populations included in the study. Increasing salinity suppressed germination of all populations; however, differences existed among populations. Seed germination was reduced with increasing salinity, and irrigated and ruderal populations exhibited higher germination than rainfed and abandoned populations (Fig 4). Salinity levels required for retarding 50% germination of irrigated, rainfed, abandoned and ruderal populations were 289.89, 209.87, 177.39, 336.57 mM, respectively (Table 5). This indicates that abandoned population was more tolerant to salinity followed by irrigated population.

**Fig 4:** The influence of different salinity levels on seed germination of *Conyza stricta* Willd. The vertical bars present standard errors of means (n = 10).

**Table 5:** Effect of different environmental conditions on seed germination of different populations of *Conyza stricta* Willd. modeled with three parametric sigmoidal equation.

Population	G_max_	T_50_	G_rate_	R^2^
**Salinity levels**				
Irrigated	89.67±3.90	289.89±13.94	-88.75±10.64	0.98
Rainfed	96.60±3.03	209.87±24.64	-103.75±14.31	0.97
Abandoned	97.32±1.22	177.39±27.19	-91.43±15.34	0.96
Ruderal	87.31±2.39	336.57±9.54	-89.18±7.38	0.99
**Osmotic potentials**				
Irrigated	91.75±3.71	0.71±0.02	-0.19±0.03	0.98
Rainfed	93.05±1.63	0.83±0.01	-0.15±0.02	0.99
Abandoned	85.46±1.88	0.82±0.02	-0.14±0.03	0.99
Ruderal	90.65±2.45	0.75±0.01	-0.18±0.02	0.99

Parameter estimates: G_max_ = maximum germination (%), T_50_ = time to reach 50% of the maximum germination (days), G_rate_ = slope of three parametric sigmoidal function fitted to model the germination of different populations of Erect horseweed. R^2^ represents the model goodness of fit.

Soil salinity is regarded as first barrier for establishment and germination of plant species [58]. Soil salinity suppresses seed germination by osmotic stress and ion inclusion. Weed species have evolved several mechanisms to tolerate salinity [58–60]. The differences in the salinity tolerance among populations are directly related to soil salinity levels of the sites of origin of the populations. Soils of abandoned and irrigated populations were saline (Table 2), which imparted better salinity tolerance than other populations. Several earlier studies have reported significant differences among weed populations for salinity tolerance [16, 17] and linked these difference either with morphological variations or soil properties.

### Osmotic potential

Seed germination of tested populations was altered by different osmotic potentials used in the study. Increasing negative osmotic potential retarded seed germination; however, differences were noted among populations. Seed germination was reduced with increasing osmotic potential with rainfed and abandoned populations exhibiting higher tolerance to increased osmotic potential (Fig 5). Osmotic potentials required for suppressing 50% germination of irrigated, rainfed, abandoned and ruderal populations were -0.71, -0.83, -0.82 and -0.75 MPa, respectively (Table 5). This indicates that rainfed and abandoned populations were more tolerant to osmotic stress.

**Fig 5:** The influence of different osmotic potentials on seed germination of *Conyza stricta* Willd. The vertical bars present standard errors of means (n = 10).

Water imbibition is an essential step of seed germination [33] and moisture uptake is reduced under negative osmotic potential. Increased osmotic potential probably caused osmotic stress, resulting in less water imbibition [33]. Lower water imbibition did not activate necessary physiological processes, resulting in low seed germination. Populations arising from rainfed and abandoned habitats exhibited higher tolerance to increasing osmotic potential. The possible reason of increased tolerance is low moisture availability at the sites of origin. Environmental conditions faced by maternal plants strongly alter germination characteristics of plant species [17]. Thus, seeds produced by the plants under low moisture availability proved more tolerant to increased osmotic stress.

### pH

Different pH levels exerted significant impact on seed germination of tested populations. Seeds of all populations were able to germinate under a broad range of pH (3–12). However, germination initially increased with increasing pH up to neutral level and then declined (Fig 6). The highest seed germination of irrigated, rainfed, abandoned and ruderal populations was recorded under 7.07, 7.03, 7.32 and 7.34 pH, respectively (Table 4).

**Fig 6:** The influence of different pH levels on seed germination of *Conyza stricta* Willd. The vertical bars present standard errors of means (n = 10).

Soil pH affects water uptake ability of plant species. The highest moisture uptake and seed germination of several weed species have been recorded under neutral pH [16, 26, 61, 62]. Slight differences among seed germination ability of different populations can be explained with differences in soil properties of seed collection sites.

### Seed burial depth

Different seed burial depths significantly influenced seedling emergence of tested populations. Seedling emergence was initially increased with increasing seed burial depth, reached to the highest level and declined sharply (Fig 7). Irrigated population exhibited higher seedling emergence than rest of the populations (Fig 7). The highest seedling emergence of irrigated, rainfed, abandoned and ruderal populations was recorded under 1.77, 1.72, 1.62 and 1.69 cm burial depths, respectively (Table 4).

**Fig 7:** The influence of different seed burial depths on seedling emergence of *Conyza stricta* Willd. The vertical bars present standard errors of means (n = 10).

Seed burial depth controls seedling emergence by soil-seed contact, moisture uptake, light availability and mechanical impedance. Deep buried seeds often face resistance due to mechanical impedance of soil. Seeds placed on surface undergo poor contact with soil, ultimately resulting in low moisture uptake. Nonetheless, surface seeds are exposed to sunlight, which results in dehydration and eventually seeds become unable to germinate. There are numerous reports indicating that seedling emergence of surface placed seeds is poor due to less moisture uptake [26, 61–63]. Deep burial lowers sunlight penetration; thus, photoblastic seeds buried at higher depths are unable to emerge. Mechanical impedance offered by the soil further aggravates the situation. Sharp decline in seedling emergence of deep buried seeds of all populations is directly linked with photoblastic nature (Fig 1). Seeds require 12-hour light dark period and deep burial did not provide required light duration for germination. Numerous studies on weed species have indicated decline in seedling emergence of deep buried seeds [16, 17, 26, 28, 61, 62]. Seedling emergence and photoblastic nature of the seeds provides an excellent seed management tactics against the species. Tillage could exploited as a weed management tactic in conservation agriculture [10]. Increasing cases of herbicide resistance weeds has forced scientists to find alternatives of herbicides, and tillage is being used to manage weeds [11]. Reducing soil seed bank is the long-term goal of tillage. Several studies have been conducted to infer the impact of tillage practices on soil seed bank and contrasting results have been reported. Studies have reported an increase [12], decrease [13] or no impact [14] of tillage on soil seed bank. Nonetheless, various studies on seed germination biology of weed species have indicated that tillage can be used to reduce soil seed bank in long run [15–17]. Thus, the result of seed burial experiments indicate that tillage can be used as a viable tool to manage *C*. *stricta*. Seed burial >4 cm depth and subsequent management of rare emerging seedlings can deplete the soil seed bank and successfully manage the species in agricultural fields.

## Conclusion

Seeds of tested population germinated under a broad range of environmental conditions, which explains the distribution of *Conyza stricta* in diverse habitats. Furthermore, the species could extend its range due to broad seed germination niche. Seeds of all populations were purely photoblastic and required 12-hour light/dark period for germination. Seedling emergence was severely retarded after 2 cm burial depth providing hope for the management of the species in agricultural habitats. Deep seed burial followed by conservational tillage can successfully manage the species in agricultural fields. However, immediate management strategies are needed for the species in other habitats.

## References

[1] LiTSC. Chinese & Related North American Herbs CRC Press; 2016 10.1201/9781420094169

[2] OttaviniD, PannacciE, OnofriA, TeiF, JensenPK. Effects of Light, Temperature, and Soil Depth on the Germination and Emergence of *Conyza canadensis* (L.) Cronq. Agronomy. 2019 10.3390/agronomy9090533

[3] TrezziMM, VidalRA, PatelF, MiottoE, DebastianiF, BalbinotAA, et al Impact of *Conyza bonariensis* density and establishment period on soyabean grain yield, yield components and economic threshold. Weed Res. 2015;55: 34–41. 10.1111/wre.12125

[4] ZinzolkerA, KigelJ, RubinB. Effects of environmental factors on the germination and flowering of *Conyza albida*, *C*. *bonariensis* and *C*. *canadensis*. Phytoparasitica. 1985;13: 229–230.

[5] WuH, WalkerS, RollinMJ, TanDKY, RobinsonG, WerthJ. Germination, persistence, and emergence of flaxleaf fleabane (*Conyza bonariensis* [L.] Cronquist). Weed Biol Manag. 2007;7: 192–199.

[6] WeaverSE. The biology of Canadian weeds. 115. *Conyza canadensis*. Can J Plant Sci. 2001;81: 867–875.

[7] LouraD, Sahil, FlorentineS, ChauhanBS. Germination ecology of hairy fleabane (*Conyza bonariensis*) and its implications for weed management. Weed Sci. 2020 10.1017/wsc.2020.28

[8] VargasL, BianchiMA, RizzardiMA, AgostinettoD, Dal MagroT. Buva (*Conyza bonariensis*) resistente ao glyphosate na região sul do Brasil. Planta Daninha. 2007;25: 573–578. 10.1590/S0100-83582007000300017

[9] AgostinettoD, VargasAAM, RuchelQ, SilvaJDG da, VargasL. Germination, viability and longevity of horseweed (*Conyza* spp.) seeds as a function of temperature and evaluation periods. Ciência Rural. 2018;48 10.1590/0103-8478cr20170687

[10] NicholsV, VerhulstN, CoxR, GovaertsB. Weed dynamics and conservation agriculture principles: A review. F Crop Res. 2015;183: 56–68. 10.1016/j.fcr.2015.07.012

[11] Heap I. The International Herbicide-Resistant Weed Database. 2020. Available: http://www.weedscience.org/Home.aspx

[12] SosnoskieLM, CardinaJ, HermsCP, KleinhenzM. Weed Seedbank Community Composition in a 35-Year-Old Tillage and Rotation Experiment. HortScience. 2004;39: 845C – 845. 10.21273/HORTSCI.39.4.845C

[13] MurphySD, ClementsDR, BelaoussoffS, KevanPG, SwantonCJ. Promotion of weed species diversity and reduction of weed seedbanks with conservation tillage and crop rotation. Weed Sci. 2006;54: 69–77. 10.1614/WS-04-125R1.1

[14] Bàrberi P, Bonari E, Mazzoncini M, García-Torres L, Benites J, Martínez-Vilela A. Weed density and composition in winter wheat as influenced by tillage systems. Conservation agriculture, a worldwide challenge. Proc of the First World Congress on Conservation Agriculture, Madrid, Spain. 2001. pp. 451–455.

[15] OzaslanC, FarooqS, OnenH, OzcanS, BukunB, GunalH. Germination Biology of Two Invasive *Physalis* Species and Implications for Their Management in Arid and Semi-arid Regions. Sci Rep. 2017;7: 16960 10.1038/s41598-017-17169-5 29208989PMC5717255

[16] ÖnenH, FarooqS, TadS, ÖzaslanC, GunalH, ChauhanBS. The Influence of Environmental Factors on Germination of Burcucumber (*Sicyos angulatus*) Seeds: Implications for Range Expansion and Management. Weed Sci. 2018;66: 494–501. 10.1017/wsc.2018.20

[17] FarooqS, OnenH, OzaslanC, BaskinCC, GunalH. Seed germination niche for common ragweed (*Ambrosia artemisiifolia* L.) populations naturalized in Turkey. South African J Bot. 2019;123: 361–371.

[18] BoscuttiF, SiguraM, GambonN, LagazioC, KrüsiBO, BonfantiP. Conservation Tillage Affects Species Composition But Not Species Diversity: A Comparative Study in Northern Italy. Environ Manage. 2014 10.1007/s00267-014-0402-z 25392019

[19] ShahzadM, FarooqM, HussainM. Weed spectrum in different wheat-based cropping systems under conservation and conventional tillage practices in Punjab, Pakistan. Soil Tillage Res. 2016;163: 71–79. 10.1016/j.still.2016.05.01228913583

[20] FarooqM, NawazA. Weed dynamics and productivity of wheat in conventional and conservation rice-based cropping systems. Soil Tillage Res. 2014;141: 1–9. 10.1016/j.still.2014.03.012

[21] Al-WahaibiLH, Al-SaleemMSM, BasudanOA, Abdel-MageedWM. Flavonoid dimers from the aerial parts of *Conyza stricta*. Biochem Syst Ecol. 2019;87: 103959 10.1016/j.bse.2019.103959

[22] AhmedM, AhmedAA. Terpenoids from *Conyza stricta*. Phytochemistry. 1990;29: 2715–2716. 10.1016/0031-9422(90)85226-6

[23] FowlerR, RockstromJ. Conservation tillage for sustainable agriculture. Soil Tillage Res. 2001;61: 93–108. 10.1016/S0167-1987(01)00181-7

[24] PittelkowCM, LiangX, LinquistBA, van GroenigenKJ, LeeJ, LundyME, et al Productivity limits and potentials of the principles of conservation agriculture. Nature. 2015;517: 365–368. 10.1038/nature13809 25337882

[25] KassamA, FriedrichT, DerpschR. Global spread of Conservation Agriculture. Int J Environ Stud. 2019 10.1080/00207233.2018.1494927

[26] AwanTH, ChauhanBS, Sta CruzPC. Influence of environmental factors on the germination of *Urena lobata* L. and its response to herbicides. PLoS One. 2014;9 10.1371/journal.pone.0090305 24658143PMC3962347

[27] ChauhanBS, JohnsonDE. Seed germination ecology of junglerice (*Echinochloa colona*): a major weed of rice. Weed Sci. 2009;57: 235–240.

[28] ChauhanBS. Germination biology of *Hibiscus tridactylites* in Australia and the implications for weed management. Sci Rep. 2016;6: 26006 10.1038/srep26006 27174752PMC4865874

[29] VidalRA, KalsingA, Goulart ICG dosR, LamegoFP, ChristoffoletiPJ. Impacto da temperatura, irradiância e profundidade das sementes na emergência e germinação de *Conyza bonariensis* e *Conyza canadensis* resistentes ao glyphosate. Planta daninha. 2007;25: 309–315.

[30] Valencia‐GredillaF, SupicicheML, ChantreGR, RecasensJ, Royo‐EsnalA. Germination behaviour of *Conyza bonariensis* to constant and alternating temperatures across different populations. Ann Appl Biol. 2020;176: 36–46. 10.1111/aab.12556

[31] KarlssonLM, MilbergP. Comparing after-ripening response and germination requirements of *Conyza canadensis* and *C*. *bonariensis* (Asteraceae) through logistic functions. Weed Res. 2007 10.1111/j.1365-3180.2007.00576.x

[32] YamashitaOM, GuimarãesSC, FigueiredoMC, de CarvalhoAMAC, MassarotoJA, KogaPS, et al Germinação de sementes de duas espécies de Conyza em função da presença ou ausência de luz e interação com a adição de nitrato e ácido giberélico no substrato. Ambiência. 2016;12: 655–666.

[33] BewleyJD, BradfordKJ, HilhorstHWM, NonogakiH. Seeds: Physiology of development, germination and dormancy, 3rd edition. Seeds: Physiology of Development, Germination and Dormancy, 3rd Edition. 2013 10.1007/978-1-4614-4693-4

[34] NandulaVK, EubankTW, PostonDH, KogerCH, ReddyKN. Factors affecting germination of horseweed (*Conyza canadensis*). Weed Sci. 2006 10.1614/ws-06-006r2.1

[35] ForcellaF, Benech ArnoldRL, SanchezR, GhersaCM. Modeling seedling emergence. F Crop Res. 2000 10.1016/S0378-4290(00)00088-5

[36] GarcíaAL, RecasensJ, ForcellaF, TorraJ, Royo-EsnalA. Hydrothermal Emergence Model for Ripgut Brome (*Bromus diandrus*). Weed Sci. 2013 10.1614/ws-d-12-00023.1

[37] Royo-EsnalA, GarcíaAL, TorraJ, ForcellaF, RecasensJ. Describing *Polygonum aviculare* emergence in different tillage systems. Weed Res. 2015 10.1111/wre.12154

[38] Zambrano-NaveaC, BastidaF, Gonzalez-AndujarJL. A hydrothermal seedling emergence model for *Conyza bonariensis*. DavisA, editor. Weed Res. 2013;53: 213–220. 10.1111/wre.12020

[39] Zambrano-NaveaC, BastidaF, Gonzalez-AndujarJL. A cohort-based stochastic model of the population dynamic and long-term management of *Conyza bonariensis* in fruiting tree crops. Crop Prot. 2016;80: 15–20. 10.1016/j.cropro.2015.10.023

[40] LazarotoCA, FleckNG, VidalRA. Biologia e ecofisiologia de buva (*Conyza bonariensis* e *Conyza canadensis*). Ciência Rural. 2008;38: 852–860.

[41] GórskiT. Germination of seeds in the shadow of plants. Physiol Plant. 1975;34: 342–346.

[42] Michael PW. Some weedy species of Amaranthus (amaranths) and Conyza/Erigeron (fleabanes) naturalised in the Asian-Pacific region. Proceedings of the 6th Asian-Pacific Weed Sci Soc Conference (Jakarta, Indonesia, 11–17 July 1977). Asian-Pacific Weed Science Society; 1977. pp. 87–95.

[43] TremmelDC, PetersonKM. Competitive subordination of a piedmont old field successional dominant by an introduced species. Am J Bot. 1983 10.2307/2443282

[44] BuhlerDD, OwenMDK. Emergence and survival of horseweed (*Conyza canadensis*). Weed Sci. 1997;45: 98–101. 10.1017/S0043174500092535

[45] ShahzadM, FarooqM, JabranK, HussainM. Impact of different crop rotations and tillage systems on weed infestation and productivity of bread wheat. Crop Prot. 2016;89: 161–169.

[46] ChauhanBS, GillG, PrestonC. Factors affecting seed germination of threehorn bedstraw (*Galium tricornutum*) in Australia. Weed Sci. 2006;54: 471–477.

[47] MichelBE, KaufmannMR. The osmotic potential of polyethylene glycol 6000. Plant Physiol. 1973;51: 914–916. 10.1104/pp.51.5.914 16658439PMC366375

[48] BarretoLC, SantosFMG, GarciaQS. Seed dormancy in Stachytarpheta species (Verbenaceae) from high-altitude sites in south-eastern Brazil. Flora Morphol Distrib Funct Ecol Plants. 2016;225: 37–44. 10.1016/j.flora.2016.09.009

[49] WellerSL, FlorentineSK, SillitoeJF, GrechCJ, McLarenDA. An investigation of the effects of stage of ensilage on *Nassella neesiana* seeds, for reducing seed viability and injury to livestock. Sci Rep. 2016;6: 22345 10.1038/srep22345 26925589PMC4772109

[50] ShapiroSS, WilkMB. An analysis of variance test for normality (complete samples). Biometrika. 1965;52: 591–611.

[51] SteelRGD, TorrieJH, DickeyD. Principles and Procedures of Statistics: a Biometrical Approach, New York McGraw-Hill; 1980.

[52] IBM SPSS Inc. SPSS Statistics for Windows IBM Corp Released 2012 2012;Version 20: 1–8.

[53] Eslami SV. Comparative germination and emergence ecology of two populations of common lambsquarters (*Chenopodium album*) from Iran and Denmark. Weed Sci. 2011;59: 90–97.

[54] LommenSTE, HallmannCA, JongejansE, ChauvelB, Leitsch-VitalosM, AleksanyanA, et al Explaining variability in the production of seed and allergenic pollen by invasive *Ambrosia artemisiifolia* across Europe. Biol Invasions. 2018;20: 1475–1491. 10.1007/s10530-017-1640-9

[55] BürgerJ, Malyshev AV., ColbachN. Populations of arable weed species show intra-specific variability in germination base temperature but not in early growth rate. PLoS One. 2020 10.1371/journal.pone.0240538 33035273PMC7546504

[56] SaeedA, HussainA, KhanMI, ArifM, MaqboolMM, MehmoodH, et al The influence of environmental factors on seed germination of *Xanthium strumarium* L.: Implications for management. PLoS One. 2020 10.1371/journal.pone.0241601 33125445PMC7598500

[57] Pamplona J deP, Souza M deF, SousaDMM, de MesquitaHC, FreitasCDM, LinsHA, et al Seed germination of Bidens subalternans DC. exposed to different environmental factors. PLoS One. 2020;15: e0233228 10.1371/journal.pone.0233228 32407422PMC7224472

[58] FarooqS, TadS, OnenH, GunalH, CaldiranU, OzaslanC. Range expansion potential of two co-occurring invasive vines to marginal habitats in Turkey. Acta Oeocologica. 2017;84: 23–33. 10.1016/j.actao.2017.08.004

[59] OnenH, FarooqS, GunalH, OzaslanC, ErdemH. Higher Tolerance to Abiotic Stresses and Soil Types May Accelerate Common Ragweed (*Ambrosia artemisiifolia*) Invasion. Weed Sci. 2017;65: 115–127. 10.1614/WS-D-16-00011.1

[60] ÖzaslanC, FarooqS, OnenH, BukunB, OzcanS, GunalH, et al Invasion Potential of Two Tropical Physalis Species in Arid and Semi-Arid Climates: Effect of Water-Salinity Stress and Soil Types on Growth and Fecundity. PLoS One. 2016;11: 1–23. 10.1371/journal.pone.0164369 27741269PMC5065205

[61] ChauhanBS, JohnsonDE. Germination ecology of Chinese sprangletop *(Leptochloa chinensis*) in the Philippines. Weed Sci. 2008;56: 820–825.

[62] MahmoodAH, FlorentineSK, ChauhanBS, McLarenDA, PalmerGC, WrightW. Influence of various environmental factors on seed germination and seedling emergence of a noxious environmental weed: green galenia (*Galenia pubescens*). Weed Sci. 2016;64: 486–494.

[63] ChauhanBS, JohnsonDE. The role of seed ecology in improving weed management strategies in the tropics. Adv Agron. 2010;105: 221–262.

